The article "Functional Imaging in Improving Children's Mental Health Based on Behavior" was published in 2022. Journal: Comput Math Methods Med.

# Functional Imaging in Improving Children's Mental Health Based on Behavior

**DOI:** 10.1155/2022/4774771

**Published:** 2022-07-16

**Authors:** Hua Li, Yuehua Lei, Tao Guo, Xiang Zhang, Hong Zhu

**Affiliations:** ^1^Chengdu Qingbaijiang Maternal and Child Health Care Hospital, Chengdu, 610300 Sichuan, China; ^2^School of Education and Psychology, Chengdu Normal University, Chengdu, 611130 Sichuan, China

## Abstract

At present, children's psychological and behavioral health care is mainly based on the doctor's observation and diagnosis. On the whole, it is inefficient, and the effect of health care cannot meet the current needs of children's behavior. Therefore, this paper uses the method of functional imaging to study the key factors of children's behavioral health care. In this paper, the structure and function of children's brain are associated with children's psychological behavior. The brain structure of 64 children in our city is detected by functional image processing, and 64 children are divided into groups according to the detection results. According to the children's performance, the children were divided into physical disorder (11 cases), emotional disorder (14 cases), cognitive disorder (12 cases), and normal group (42 cases). Among them, 3 cases had three kinds of disorders, 6 cases had both emotional and cognitive disorders, 7 cases had physical and emotional disorders, and 5 cases had physical and cognitive disorders. In this paper, according to the research data of functional imaging on different levels of children's brain, we use computer to model and simulate through digital conversion technology, draw the neural network Atlas of children's psychological behavior, compare the children's representation and image characteristics according to functional imaging, and then, study the relationship between children's signs and images, to make a plan for improving children's psychological behavior health care. The study shows that in the above different groups, the linear correlation between the functional imaging results and the representation of 22 abnormal children is 98%, and the fuzzy deviation is only 3.52%, which indicates that functional imaging can be used as the basic judgment basis in improving children's psychological and behavioral health care and can predict and reasonably prevent children's potential psychological behavior according to the images.

## 1. Introduction

The attitude and actions of parents have a significant influence on their children's outside activities and depressed time. One of the primary causes of children's mental problems in developing nations is a lack of knowledge among parents or guardians about how to improve mental health and where to get adequate mental health treatment. Despite the fact that the school mental health management program has increased the prevalence of ametropia diagnosis, many children with ametropia continue to fail to meet the standards of psychological illnesses.

Joan et al. put forward a comprehensive multilevel pyramid (four level management) mental health management scheme, which aims to provide cost-effective mental health services for children aged 0-15 years in the project area and help them take intervention measures [1]. Jaffee analyzed the lifestyle factors related to the progress of mental disorders in Japanese third-grade primary school students. High weight, parents' mental disorders, and Western food eating habits were associated with the increased prevalence of mental disorders [2]. Giessen and Bgels reported the relationship between mental disorders and BMI, and children with mental disorders had a higher risk of mental disorders [3]. On this basis, Panagiotaki et al. put forward the concept of human brain connectomics in 2020, believing that the information processing of the brain has the characteristics of network [4]. Fong et al. used the task design of children's psychological and behavioral health care during fMRI scanning and found that children's psychological and behavioral health care can effectively reduce the functional activities of limbic system of healthy subjects [5]. Chua et al.'s research shows that parents' untimely behavior of seeking mental health for their children is the result of lack of mental health knowledge [6].

Thomas et al. randomly selected 173 parents studying in Swaziland public schools to conduct a questionnaire survey on children's psychological health care. The results showed that 104 (60.1%) parents had never taken their children for psychological examination, 69 (31.7%) thought their children were in good psychology, and 97 (53.1%) parents said they knew nothing about children's psychological diseases [7]. Resnikoff et al.'s survey shows that parents of children with mental disorders under 12 years old have significantly lower awareness of basic mental health knowledge such as mental health exercises, correct reading and writing posture, controlling the time of using TV or mobile phone, and using mental health than parents of children with mental disorders of the same age [8]. Bourne found that children with shorter sleep time were more likely to have mental disorders [9]. Among 460 students aged 11-15 randomly recruited by Das T, 78.7% (362/460) were followed up. After 3-4 months of psychological distribution, 25.4% (92/362) had no psychological disorder [10]. The above studies show that the network connections between microscale neurons, mesoscale neuronal clusters, and macroscale brain regions are characterized by the combination of simple connections and efficient and economic topological connections. However, there is a lack of clinical experimental data of medical imaging, and the relationship between children's psychological behavior cannot be studied from the physiological point of view.

The functional imaging approach was utilized in this work to investigate the essential determinants of children's behavioral health care. The form and function of children's brains are linked to their psychological behavior in this research. The functional image processing detects the brain structure of 64 children in our city, and the 64 children are separated into groups based on the detection findings. In this paper, we use computer to model and simulate through digital conversion technology, draw the neural network Atlas of children's psychological behavior, compare the children's representation and image characteristics according to functional imaging, and then, study the relationship between children's signs and images, in order to make a plan for improving children's IQ.

## 2. Children's Psychological and Behavioral Health Care and Functional Image Processing Methods

### 2.1. Children's Psychological and Physical Activities

Physical activity is defined as any body activity that results in energy consumption and is participated by skeletal muscles. Physical activity can accelerate heart rate and sweat [11]. Physical exercise is a purposeful, planned, structured, and organized physical activity, repeated training to improve and maintain physical condition [12]. RCT studies of preterm infants suggest that physical activity contributes to weight gain, linear growth, and bone mineralization. Research on physical activity in infants and young children shows that physical activity not only contributes to weight and length growth but also plays an important role in the formation of bone, muscle, and body mass tissue, and this healthy physical model can last until adulthood [13]. According to the review of 19 cohort studies on children, physical activity is very important for the formation of peak bone mass, especially in the peak growth period, but it does not affect height [14]. The brain test of children is shown in Figure 1.

It is suggested that children's physical exercise contributes to the health of bone and muscle tissue, but the effect on height is uncertain. Sleep is necessary for children's growth. There is pulse release of growth hormone during slow wave sleep. Chronic sleep deprivation in children may affect linear growth, but this hypothesis has not been systematically tested [15]. Many studies on sleep have found that short sleep time in children is associated with increased risk of psychological disorders [16]. In conclusion, proper physical activity/physical exercise and adequate sleep are beneficial to children's physical health, including the health of bones and muscles, the distribution of body mass tissue, and the reduction of the risk of psychological disorders [17]. However, the effect on height is lack of sufficient evidence. There was no significant correlation between sleep time and bedtime and the progress of mental disorders and mental axis elongation [18]. The reason is not clear. Regular sleep can ensure normal circadian rhythm and growth and development. Insufficient sleep may have a negative impact on mental eye growth by interfering with mental rhythm [19].

### 2.2. Psychological and Behavioral Health Care

The main complication of psychological and behavioral health care is aortic rupture. It is estimated that there are 150000-200000 deaths associated with abdominal aortic aneurysm every year in the world [20]. Since the 1970s, many studies have proved that the diameter of abdominal aorta is related to the rupture of psychological and behavioral health care. Therefore, the maximum diameter of psychological and behavioral health care (effectively measured by diagnostic ultrasound) has become the main factor determining the treatment options of patients [21]. Current guidelines recommend that smaller (diameter of psychological and behavioral care <50 mm for women and <55 mm for men) and asymptomatic psychological and behavioral care should be managed by interval monitoring imaging, while larger or symptomatic psychological and behavioral care should be managed by open surgery or endovascular surgery [22]. Therefore, effective screening and evaluation means are very important for the correct detection and treatment of psychological and behavioral health care [23]. At present, MRI (magnetic resonance imaging) is used in the diagnosis of psychological and behavioral health care, but abdominal ultrasound is still the preferred imaging method. Ultrasound imaging is a relatively cheap, accurate, and reliable method to detect psychological and behavioral health care, with 95% sensitivity and nearly 100% specificity [24].

When the tension on the abdominal aorta wall surpasses its strength, that is, when the abdominal aorta wall cannot withstand the stress, the psychological and behavioral health care might burst. Although the specific mechanism of psychological and behavioral health care disorders is unknown, inflammation, extracellular matrix remodeling, angiogenesis, and thrombosis all have a role in the pathogenesis of psychological and behavioral health care disorders. These biological processes cause elastin degradation and collagen changes, reducing the strength and elasticity of the abdominal aorta [25]. The process of mechanical alterations and rupture of the abdominal aortic wall, however, remains unknown.

### 2.3. Functional Image Processing Algorithm

However, diameter can neither represent growth rate nor rupture risk nor reflect the complexity of aneurysm blood flow

(1) $$\begin{array}{c} W\left(Ai,Aj\right)=\left[\frac{\log\left(\left|x_{A_{i}}-a_{A_{j}}\right|/w_{A_{j}}\right),\log\left(\left|y_{A_{i}}-y_{A_{j}}\right|/h_{A_{j}}\right)}{\log\left(w_{A_{i}}/w_{A_{j}}\right),\log\left(h_{A_{i}}/h_{A_{j}}\right)}\right],\\ W\left(\log s_{j}\right)=\underset{i}{\sum }c_{ij}u_{\left(j\left|i\right.\right)}. \end{array}$$

Therefore, new indicators are needed to help detect high-risk aneurysms that do not meet the current diameter-based treatment threshold and to avoid intervention for patients with large but low-risk aneurysms. The linear relationship between intervention and *D* was as follows:

(2) $$\begin{array}{c} D=\overset{n}{\underset{\delta =1}{\sum }}Z_{ikjl}\left(\varepsilon \right),\\ Z_{t}=\sigma \left(w_{r}x_{t}+u_{r}h_{t-1}+Z_{r}\right). \end{array}$$

The complex geometry of psychological and behavioral health care may form blood flow patterns such as recirculation zone, vortex, and stagnation zone, which may affect the growth and rupture risk of psychological and behavioral health care:

(3) $$\begin{array}{c} {\frac{D}{Z}}_{t}=\tanh\left(w_{c}x_{t}+u_{c}\left(r_{t}\Theta h_{t-1}\right)+b_{c}\right),\\ \text{MR}{\text{I}}_{t}=z_{t}\Theta H_{t-1}+\left(1-z_{t}\right)\Theta H_{t}. \end{array}$$

The noninvasive medical imaging methods that can locate and quantify these areas will be of great significance in optimizing treatment. With the advent of MRI technology, MRI has many advantages over CT in the study of morphology and hemodynamics of cardiovascular diseases:

(4) $$\begin{array}{c} \text{CT}=\overset{N}{\underset{i,j}{\sum }}f\left(X_{ij}\right){\left(v_{i}^{T}v_{j}+b_{i}+b_{j}-\log\left(X_{ij}\right)\right)}^{2},\\ X_{ij}=\frac{X_{i}/X_{j}}{\log\left(\left|x_{A_{i}}-a_{A_{j}}\right|/w_{A_{j}}\right)}. \end{array}$$

The changes of blood flow pattern and hemodynamics may play an important role in predicting the complications of psychological and behavioral health care and judging the prognosis. However, its disadvantage is that two-dimensional phase contrast MRI is limited to imaging a single 2D plane:

(5) $$\begin{array}{c} {\frac{\left|y_{A_{i}}-y_{A_{j}}\right|}{h_{A_{j}}}}_{t}=\sigma \left(W_{0}\cdot h_{t}\right),\\ \sigma_{ikjl}=\left\{\begin{array}{cc} \frac{n}{\Delta_{ikjl}}\sqrt{\overset{n}{\underset{s=1}{\sum }}{\left(x_{ik}\left(\varepsilon \right)-x_{jl}\left(\varepsilon \right)\right)}^{2}\Delta_{ikjl}\left(\varepsilon \right)}, & \Delta_{ikjl}>0,\\ 0, & \Delta_{ikjl}<0. \end{array}\right. \end{array}$$

The improved four-dimensional flow sensitive mapping (4D flow MRI) provides a direct, noninvasive measurement of cardiovascular hemodynamics, which can visualize and quantify the blood stasis of psychological and behavioral health care:

(6) $$\begin{array}{c} E_{1}^{ij}=\frac{\cos\left(S_{1}^{i},S_{2}^{j}\right)}{\left(1-z_{t}\right)\Theta H_{t}}, \end{array}$$

(7) $$\begin{array}{c} {\frac{z}{E}}_{t}=\sigma \left(w_{z}x_{t}+u_{z}h_{t-1}+b_{z}\right). \end{array}$$

This image-based quantification of blood flow stagnation may provide another way for risk stratification of psychological and behavioral health care or prediction of the growth of intracavitary thrombosis. 4D flow MRI is a phase contrast technique, which is used to estimate wall shear stress from time-resolved three-dimensional velocity profile. It can accurately measure blood flow velocity flow, forward blood flow *a*, backward blood flow *Z*, blood flow morphology, and reflux fraction:

(8) $$\begin{array}{c} \text{Flow}{\left(w_{z}x_{t}+u_{z}h_{t-1}+b_{z}\right)}_{ij}=\frac{e^{b_{ij}}\log\left(\left|y_{A_{i}}-y_{A_{j}}\right|/h_{A_{j}}\right)}{\sum_{k}e^{b_{ik}}}+\log\left(\frac{h_{A_{i}}}{h_{A_{j}}}\right),\\ {\frac{h_{A_{i}}}{h_{A_{j}}}}_{\left(j\left|i\right.\right)}=w_{ij}\frac{e^{b_{ij}}\log{\left(\left|y_{A_{i}}-y_{A_{j}}\right|/h_{A_{j}}\right)}_{i}}{\left(w_{r}x_{t}+u_{r}h_{t-1}+Z_{r}\right)},\\ A_{t2}=\frac{\left(w_{1}^{2},w_{2}^{2},w_{3}^{2},w_{4}^{2},w_{5}^{2}\right)}{e^{b_{ij}}\log\left(\left|y_{A_{i}}-y_{A_{j}}\right|/h_{A_{j}}\right)}. \end{array}$$

However, more research is needed to understand the relationship between 4D blood flow parameters and arterial wall in different disease states:

(9) $$\begin{array}{c} \log\left(\frac{\left|y_{A_{i}}-y_{A_{j}}\right|}{h_{A_{j}}}\right)\left(a,b\right)=\frac{a\cdot b}{\left|a\right|*\left|b\right|}. \end{array}$$

The diameter of psychological behavior health care is still the most definite factor in the risk of psychological behavior health care disorder. The rapid development of molecular imaging technology provides great hope for better monitoring the progress of diseases in vivo. High-resolution ultrasound and functional and molecular imaging techniques can be used to evaluate ZD index, such as hemodynamics, aortic wall dynamics, circumferential strain, wall stiffness, vascular calcification, vascular wall inflammation, and extracellular matrix degradation:

(10) $$\begin{array}{c} \text{ZD}\left(k\right)=\frac{{\left\|k\right\|}^{2}}{1+{\left\|k\right\|}^{2}}\frac{k}{\left\|k\right\|},\\ k_{j}=\frac{E\left(s_{j}\right)}{\sigma \left(w_{z}x_{t}+u_{z}h_{t-1}+b_{z}\right)}+\cos\left(S_{1}^{i},S_{2}^{j}\right). \end{array}$$

In order to assess the risk of psychological and behavioral health care disorders, it is not clear which imaging method will replace CT and color Doppler ultrasound. The application of new molecular imaging is expected to improve the understanding of the biological mechanism of psychological and behavioral health care disorders. In the future, the method to evaluate psychological and behavioral health care will be the combination of anatomy and molecular imaging, such as the PET-CT imaging system including MRI under study. According to the literature, PET-MRI hybrid imaging can shorten the scanning time:

(11) $$\begin{array}{c} \text{PET}‐\text{MR}{\text{I}}_{t2}\left[i\right]=\underset{j}{\sum }\cos\left(w_{j}^{1},w_{i}^{2}\right),\\ T_{t2}=\frac{\sum_{j}\cos\left(w_{j}^{1},w_{i}^{2}\right)}{\left(v_{i}^{T}v_{j}+b_{i}+b_{j}-\log\left(X_{ij}\right.\right)}. \end{array}$$

The seamless coregistration of images obtained by different modes allows simultaneous evaluation of multiple imaging probes. This combined imaging provides great potential for better understanding of disease progression in vivo and may provide a means for better predicting psychological and behavioral health care disorders and developing specific drug therapy. It is expected that with the efforts of medical workers, the use of artificial intelligence will completely change the management and risk prediction of psychological and behavioral health care. With the deepening of neuroscience research, people gradually realize that the realization of brain specific functional activities is not based on isolated brain regions or a single mass, but by the coordination and integration of multiple brain regions.

## 3. Children's Behavior Health Care

### 3.1. Research Methods

The functional imaging approach was utilized in this work to investigate the essential determinants of children's behavioral health care. The form and function of children's brains are linked to their psychological behavior in this research. The functional image processing detects the brain structure of 64 children in our city, and the 64 children are separated into groups based on the detection findings. The youngsters were separated into four groups based on their performance: physical disorder (11 instances), emotional disorder (14 cases), cognitive disorder (12 cases), and normal (42 cases). Three of them had three types of problems, six had both emotional and cognitive disorders, seven had physical and emotional disorders, and five had both physical and cognitive disorders. In this paper, we use computer to model and simulate through digital conversion technology, draw the neural network Atlas of children's psychological behavior, compare the children's representation and image characteristics according to functional imaging, and then, study the relationship between children's signs and images, in order to make a plan for improving children's IQ.

### 3.2. Experimental Design

In this study, functional imaging was used to study the body composition of 3-8-year-old children in this city. The results showed that the body weight, BMI, fat free weight, body water, and basal metabolic rate of boys were higher than those of girls, while the body fat rate was lower than that of girls. There was no significant difference in height and body fat content between different gender groups. In the analysis of body composition of 64 children aged 5-7 years, the fat percentage and body fat content of girls were higher than boys. In this study, BMI and body water content of preschool boys were higher than those of girls, while fat content and body fat rate were lower than those of girls. The body composition analysis of preschool children showed that the body fat rate of girls was significantly higher than that of boys, but there was no significant difference in body fat, body moisture, BMI, and basal metabolism between the two groups. The body fat content of Chinese children is higher than that of Caucasian and Japanese children, and the change pattern of body composition is related to age and gender. The change pattern of body composition of Chinese boys and girls is different from that of Korean children. Therefore, there are regional differences in body composition of children of different genders. The output framework of psychological and behavioral health monitoring is shown in Figure 2.

Under this framework, we have carried out a large number of basic researches on the pathological characteristics of the disease center and the neural effects of intervention. These researches have further expanded the brain network abnormalities of Alzheimer's disease, depression, and other diseases from the perspectives of brain functional connectivity, structural connectivity, topological properties, etc., as well as the effects of transcranial magnetic stimulation (TMS), cognitive impairment, and so on, objective to understand the effect targets of new clinical techniques such as deep electrical stimulation. With the development of acupuncture and moxibustion multidisciplinary and neuroimaging of children's psychological and behavioral health care, the network analysis method based on brain connectomics is more and more widely used, and people's understanding of the regulatory effect of children's psychological and behavioral health care network is also deepening.

## 4. Results and Discussion

### 4.1. Imaging Analysis of Children's Psychological and Behavioral Health Care Function

As shown in Figure 3, biomechanical factors are the most important factors of psychological and behavioral health care disorders. The pathophysiology and biomechanics of psychological and behavioral health care disorders are much more complex than simple aneurysm diameter. The biomechanical properties of aortic wall are believed to depend on the composition and structure of aortic extracellular matrix. Aortic wall stress and aortic wall strength have an important influence on the biomechanics of psychological and behavioral health care disorders. Therefore, many studies have been devoted to explore the biomechanical relationship between aortic wall stress and aortic wall strength and the risk of psychological and behavioral health care disorders. The finite element model provides the structural analysis of the mechanical wall stress of complex aortic shape with different characteristics (i.e., different aortic wall thickness, the presence of intraluminal thrombus, and calcification). The following will elaborate the biomechanical factors of psychological and behavioral health care disorders from four aspects: aortic compliance, aortic peak wall stress, aortic wall calcification, and hemodynamics.

As shown in Figure 4, the higher the aortic wall calcification score measured from the CT image, the greater the risk of psychological and behavioral health care disorders. Microcalcification is associated with an increased risk of atherosclerotic plaque rupture, as well as an increased rate of psychological and behavioral health care expansion. Imaging used fluorine-18-labeled NaF PET-CT, CT angiography, and aortic wall calcification score to quantify active calcification. In order to solve the role of aortic wall calcification in psychological and behavioral health care disorders, more large-scale studies are needed to evaluate.

As shown in Figure 5, gender differences in the risk of psychobehavioral health care disorders may be caused not only by physiological factors (such as LDL and sex hormones), but also by anatomical factors (such as body size and aortic diameter). The hemodynamic characteristics of arteries are obviously affected by the geometric shape of arteries. Female psychological behavior health care has more complex geometric structure than male psychological behavior health care (especially the different curvature of psychological behavior health care center line). Morphological differences may lead to different hemodynamic environment, thus increasing the risk of female psychological behavior health care disorders. Hemodynamic factors play an important role in the growth and rupture of psychological and behavioral health care. The wall shear stress directly felt by endothelial cells on the lumen not only regulates vascular tension but also drives vascular remodeling; the final rupture of psychological and behavioral health care is also considered to be the result of biodegradation of arterial wall and hemodynamic forces (including wall shear stress and blood pressure).

As shown in Table 1, children's psychological and behavioral health care is a three-dimensional fibrin structure containing cholesterol crystals, which is usually composed of lumen layer, middle layer, and proximal lumen layer. The middle layer includes liquid tubules. It is usually considered as a mechanical pad, which can reduce the wall stress of psychological and behavioral health care through shielding effect, so that psychological and behavioral health care can bear greater stress without rupture; this further proves that the hemodynamics of male psychological and behavioral health care is easier to maintain the stability of psychological and behavioral health care. It may be related to the local family environment, early childhood education, and higher level of nutrition and health care. At present, BMI is an internationally recognized screening standard for mental disorders and overweight, but BMI cannot reflect the proportion of body moisture, fat-free weight, muscle mass, etc.; body composition analysis can further assess the risk of mental disorders.

As shown in Table 2, early comprehensive intervention in weight control makes body composition suitable, which can control psychological disorders and reduce the incidence rate of related diseases. With the increase of BMI, the body fat content, body fat percentage, and fat-free body weight of boys and girls increased gradually. In this study, there is a high consistency between PBF and BMI in the evaluation of overweight and mental disorders in children, but PBF has a high detection rate of overweight and mental disorders. Compared with BMI evaluation, age in PBF evaluation was significantly earlier, which had a better warning effect on psychological disorders.

As shown in Figure 6, the use of new imaging methods can promote the prediction and understanding of psychological and behavioral health care disorders. The following is a review of the latest imaging detection methods, including high-resolution ultrasound, functional and molecular imaging, and phase contrast magnetic resonance imaging. The latest imaging technology can more accurately assess the risk of psychological and behavioral health care disorders. In vitro morphometric assessment of psychobehavioral health care has many limitations, such as the inability to measure aortic diameter at maximum dilation. Ultrasound is the main technology of psychological and behavioral health screening and evaluation. Because of its high feasibility, easy operation, and real-time noninvasive imaging ability, ultrasound can accurately evaluate psychological and behavioral health in vivo.

As shown in Figure 7, compared with traditional ultrasound, the main advantage of high-resolution ultrasound is high image quality. Compared with traditional 20 kHz frequency probe, high-resolution ultrasound usually uses 20~100 MHz frequency probe, and the resolution of high-resolution ultrasound is as high as 30% *μ*m. The diameter measurement can be repeated, and the transverse imaging (short axis) and longitudinal imaging (long axis) of aorta can be performed. The system also allows the construction of three-dimensional data to better display aneurysms from different angles and planes. Other functional modules of high-resolution ultrasound, such as color Doppler mode and electrocardiogram, allow the assessment of additional parameters, thus helping to assess the risk of rupture in functional imaging. Ultrasound was also used to assess fluid dynamics (flow pattern, flow velocity, and aortic volume), aortic wall dynamics (displacement ratio, wall thickness, and radial wall velocity), circumferential strain, wall stiffness, and vascular calcification. Although noninvasive 3D ultrasound is used to improve the risk assessment of psychobehavioral health care disorders by assessing peak wall stress and aortic stiffness in healthy volunteers and patients with psychobehavioral health care during follow-up, ongoing clinical studies are needed to determine the feasibility of evaluating these results in relation to psychobehavioral health care disorders.

The measurement of the change of internal volume caused by the change of intravascular pressure is shown in Table 3, which is mainly determined by the elastic component of aortic wall. The aortic wall is considered to be expandable and compliant, and a small change in pressure in the lumen leads to a large change in volume. A prospective study of 210 patients with psychological and behavioral health care showed that the greater the aortic dilation, the higher the risk of psychological and behavioral health care disorders. After adjusting for age, gender, psychological, and behavioral health care diameter, blood pressure, and other risk factors, aortic dilation was independently associated with psychological and behavioral health care disorders. Therefore, it is necessary to have an accurate method to measure aortic distensibility in routine practice.

As shown in Table 4, the potential risk of metabolic syndrome in children, such as mental disorders and insulin resistance, is also one of the predictors of high risk of mental disorders, cardiovascular disease, and metabolic syndrome in adults. According to the change trend of BMI, the age of children in this study is about 5 years old, which is roughly consistent with the foreign and domestic studies. According to the change trend of fat content, the fat content of both boys and girls in this study increased with age, and the age was advanced to about 3 years old, suggesting that the risk of future psychological disorders in this population may be higher. Therefore, the prevention of children's psychological disorders needs to be advanced not only to primary and secondary schools but also to kindergartens.

As shown in Figure 8, functional and molecular imaging uses biomarkers or molecular tracers for functional imaging to assess molecular changes in the body. It provides a new way to study the mechanism of psychological and behavioral health care disorders in vivo. The use of isotope labeled targeted collagen, monocytes/macrophages, and matrix metalloproteinases can provide a method to monitor the risk of psychobehavioral health care disorders. Molecular MRI was used to evaluate inflammation and elastase activity. Specifically, in the psychological behavior model, macrophage-specific iron oxide probe and elastin-specific gadolinium probe were used to evaluate inflammation and elastase activity. This imaging was consistent with in vitro histology and could predict psychological behavior disorders.

As shown in Figure 9, ultrasmall superparamagnetic iron oxide particle- (USPIO-) enhanced MRI can detect cellular inflammation. USPIO-enhanced MRI is a new method to identify aortic parietal cell inflammation in patients with psychological and behavioral health care. It can predict the growth rate and clinical prognosis of aneurysms, but it is not an independent predictor. PET-CT is a common method in tumor diagnosis, which has been reported to successfully locate and quantify monocytes/macrophages in psychological and behavioral health care of patients. Fluoro-18-fluorodeoxyglucose (18F-FDG) is a commonly used radiotracer in clinic, which is used in high metabolic activity sites such as inflammation. 18F-FDG uptake is associated with psychobehavioral care and progression of thoracic aortic aneurysm. There is no convincing evidence that 18F-FDG or USPIO intake can reliably predict the growth or disruption of psychobehavioral care.

As shown in Figure 10, in the above different groups, the linear correlation between the results of functional imaging and the representation of 22 abnormal children was 98%, and the fuzzy deviation was only 3.52%, which indicated that functional imaging could be used as the basic judgment basis in improving children's psychological and behavioral health care and could predict and reasonably prevent children's potential psychological behavior according to the images.

### 4.2. Discussion

As a key technology of time connective omics, dynamic network analysis can provide a new perspective to study the integration mode of brain network in minute and second time scales, which is very suitable for the characteristics of neuroimaging research on children's psychological and behavioral health care. It is expected to become a new method to deeply explain the dynamic changes of brain network integration mode under the burden of children's psychological and behavioral health care and to further reveal the dynamic characteristics of children's psychological and behavioral health care network regulation. The second is to introduce more experimental paradigms. Different from animal experiments, inhibitors and agonists can be used to specifically study the targeted and conditional regulation of interventions. The neuroimaging research of children's psychological and behavioral health care based on clinical practice cannot achieve the blocking or stimulation of specific brain function activities. Therefore, the future neuroimaging research of children's psychological and behavioral health care can be combined with transcranial magnetic stimulation, in order to study the targeted and conditional characteristics of children's psychological and behavioral health care network regulation on the basis of specific activation or inhibition of functional activity in specific brain regions and further improve the research evidence chain. In addition, the introduction of machine learning method makes the research of neuroimaging change from the traditional paradigm based on univariate group level to the paradigm based on multivariable individual level, which provides a promising method to study the individual network regulation effect of children's psychological and behavioral health care and help children's psychological and behavioral health care precision medicine, which is also worthy of attention in future research, in order to accurately discuss the conditional characteristics of brain network regulation effect of children's psychological and behavioral health care from the individual level.

This paper puts forward that schools and parents should actively cooperate to find out the specific reasons why children with mental disorders do not admire mental disorders and improve their compliance with mental disorders. A new study analyzes the relationship between psychological disorders and the development of unhealthy psychology in children and adolescents. Psychological impairment may lead to loneliness, anxiety, even depression, and other psychological problems in the process of growing up. This also provides a perspective worthy of attention in the process of prevention and control of mental disorders of children and adolescents, which not only needs scientific research and exploration of the disease itself but also needs to protect the mental health of children with mental disorders.

## 5. Conclusions

The current neuroimaging research on children's psychological and behavioral health care has gradually shifted from focusing on the local functional activities of the brain to focusing on the integration of the overall structure and function of the brain. Understanding the central integration mode of children's psychological and behavioral health care from the perspective of brain network regulation is an important direction of neuroimaging research on children's psychological and behavioral health care. Combined with the current research status in this field and the previous research of the team, the targeted, conditional, and dynamic characteristics of the brain network regulatory effect of children's psychological and behavioral health care were preliminarily extracted. In order to have a more comprehensive and in-depth understanding of the network regulation effect characteristics of children's psychological and behavioral health care, future research can be deepened from the following aspects. The first is the application of new scanning methods and network analysis methods. At present, the research on network regulation of children's psychological and behavioral health care is basically based on magnetic resonance scanning. The follow-up research can combine magnetic resonance with EEG, near-infrared spectroscopy, and other high temporal resolution scanning methods to carry out multimodal data acquisition across devices, so as to further enrich the temporal dimension information while ensuring the high spatial resolution of magnetic resonance and to understand the network regulation effect of children's psychological and behavioral health care from multiple dimensions. In terms of analysis method, this analysis method has some limitations. Therefore, it is expected that there will be more research on children's psychological and behavioral health brain network based on causal model, complex network, dynamic model, high-order network, and other advanced algorithms in the future, to promote the improvement of research level in this field.

## Figures and Tables

**Figure 1:** Children's mental and behavioral health care monitoring sites.

**Figure 2:** Psychological health care monitoring output framework.

**Figure 3:** Critical factors in the breakdown of mental and behavioral health care.

**Figure 4:** Aortic wall calcification score.

**Figure 5:** Gender differences in the risk of mental and behavioral health care breakdown.

**Figure 6:** Prediction and recognition of mental and behavioral health care disorders.

**Figure 7:** Children's three-dimensional data.

**Figure 8:** Psychological health care breakdown risk.

**Figure 9:** High-resolution ultrasound image processing effect.

**Figure 10:** Linear correlation between test results and characterization.

**Table 1:** Wall stress for behavioral health.

Item	Aortic volume	Psychology	Flow pattern	Flow rate	Frequency
Biology	1.85	1.68	1.44	2.87	3.22
Image	4.71	4.11	4.42	2.11	3.56
Fuzzy bias	5.15	5	2.13	3.52	4.6
Linear	3.23	2.53	2.16	4.69	2.73
Function	2.45	6.07	5.57	4.84	6.79

**Table 2:** Mental disorders and reduce the incidence of related diseases.

Item	Biology	Image quality	Fuzzy bias	Linear correlation	Function image
Aortic volume	1.73	2.72	1.47	1.44	2.62
Psychology	5.8	3.73	2.77	2.62	4.62
Flow pattern	5.25	5.94	4.16	2.19	4.3
Flow rate	4.53	1.23	4.3	1.99	1.65
Frequency	4.65	6.14	4.49	1.89	5.86
Probe	1.2	5.44	1.28	6.23	5.68

**Table 3:** Internal volume of a blood vessel caused by changes in intravascular pressure.

Item	Biology	Image quality	Frequency probe	Flow rate	Aortic volume
Fuzzy bias	4.59	4.82	2.55	3.03	2.22
Linear	4.7	4.99	5.47	4.47	4.64
Function image	2.73	3.98	1.08	1.06	3.13
Characterization	5.8	5.11	1.51	5.92	6.54

**Table 4:** Psychological disorders and insulin resistance in children.

Item	Fuzzy bias	Linear correlation	Function image	Characterization
Biology	2.57	1.02	3.37	1.01
Image quality	3.84	5.76	2.6	5.05
Frequency probe	3.15	2.2	5.91	5.68
Flow pattern	1.48	1.27	2.08	2.3
Flow rate	2.5	6	3.03	4.12

## Data Availability

All of the data in this article is actually available.
